The article "Effect of Acupuncture on Simple Obesity and Serum Levels of Prostaglandin E and Leptin in Sprague-Dawley Rats" was published in 2021. Journal: Comput Math Methods Med.

# Effect of Acupuncture on Simple Obesity and Serum Levels of Prostaglandin E and Leptin in Sprague-Dawley Rats

**DOI:** 10.1155/2021/6730274

**Published:** 2021-10-04

**Authors:** Xiaomin Li, Zijian Wu, Yenong Chen, Ronglin Cai, Zhizhen Wang

**Affiliations:** ^1^Department of Traditional Chinese Medicine II Ward, Huaibei People's Hospital, Huaibei, 235000 Anhui Province, China; ^2^Institute of Acupuncture and Meridians, Anhui University of Chinese Medicine, Hefei, 230038 Anhui Province, China

## Abstract

**Aim:**

The study is aimed at investigating the curative effect of acupuncture on simple obesity and its influence on serum levels of prostaglandin E and leptin in Sprague-Dawley (SD) rats.

**Methods:**

In the study, there are 50 male SD rats. We took 10 as healthy controls and fed 40 with a diet of high fat for 8 weeks. After the 40 rat model was established successfully, we fed 10 rats in the model group with a normal diet and treated 10 rats in the acupuncture group by acupuncture. During the experiment, the body fat and body length of rats were measured weekly, and Lee's index was calculated. After the treatment, the levels of leptin, prostaglandin E, C-reactive protein (CRP), triacylglycerol (TG), cholesterol (CHO), low-density lipoprotein (LDL), and high-density lipoprotein (HDL) were detected, and the liver fat morphology was observed by electron microscope.

**Results:**

Acupuncture significantly downregulated the serum levels of CRP, TG, CHO, LDL, leptin, and prostaglandin E and upregulated the serum levels of HDL in rats with simple obesity.

**Conclusion:**

On basis of these results, it was found that acupuncture could boost fat metabolism and weight loss by inhibiting the production of leptin and prostaglandin E.

## 1. Introduction

Obesity is a complex disease that is closely related to many other diseases [1]. There are 650 million obese adults in the world, and 40% of adults in the United States are obese [2]. As one of the largest public health problems worldwide, obesity can not only lead to serious health problems but also affect the quality of life, social activities, and mental activities, leading to a heavy burden on families, patients, and the public health system. Obesity occurs when the energy intake is greater than the energy consumption and the excess energy is stored in the body in the form of fat. The condition is called obesity when the body fat content reaches a certain level [3]. There are many different interventions for obesity, including lifestyle intervention, surgery, and drug therapy. All of these have advantages and disadvantages, but unhealthy weight control behaviors may lead to many health problems [4–6].

The article "Effect of Acupuncture on Simple Obesity and Serum Levels of Prostaglandin E and Leptin in Sprague-Dawley Rats" was published in 2021. Journal: Comput Math Methods Med.

Although there are many treatment methods for simple obesity, including diet, exercise, weight-loss drug therapies, and surgical removal of fat, these methods have different degrees of adverse effects [7]. Acupuncture has a good therapeutic effect on obesity [8]. Acupuncture is a widely used medical system that has existed for thousands of years. It is becoming more and more popular in western medicine [9]. Many studies have shown that its mechanism of action can be explained in biomedical terms. During the acupuncture process, many transmitters and regulators were released, including beta-endorphin, serotonin, substance P, interleukins, and calcitonin gene-related peptide [10]. Therefore, acupuncture can be used in a variety of clinical situations. It is thought that the increased satiety center excitability in the hypothalamus ventromedial nuclei after acupuncture application can be conducive to body weight loss in obese people. Immune regulation and hormone secretion may also be involved in this process [11]. In animal models, acupuncture targeting SIRT1 in the arcuate nucleus of the hypothalamus can improve obesity in insulin-resistant rats induced by a high-fat diet through anorexia effects [12].

In the present study, before and after acupuncture treatment, we measured the serum levels of leptin, prostaglandin E, and hormones in SD rats with simple obesity to explore the possible mechanism of acupuncture during the process of treating obesity.

## 2. Materials and Methods

### 2.1. Animals

Fifty 3-month-old SPF-SD male rats (weighing approximately 200 g) were purchased from the Henan Experimental Animal Center, China. We offered food and water ad libitum. After 7 days of adaptive feeding, the rat models were prepared. The rats were fed at the Acupuncture Institute of the Anhui University of Chinese Medicine. We maintained the rats on a 12 h light-dark cycle in an environment with a humidity of 30-50% and a temperature of 20-24°C.

### 2.2. Experimental Equipment

The following devices and equipment were used: Huatuo brand filiform needle (Suzhou Medical Supplies Co., Ltd.), rat localizer and electroacupuncture therapeutic instrument (Beijing Huayunante Technology Co., Ltd.), electronic balance (Germany Saiduolis Co., Ltd.); MD-100 automatic biochemical analyser (Beijing Perlong Technology Co., Ltd.), RT-6000 microplate reader (Redu), UV-1800 ultraviolet visible spectrophotometer (Shanghai Jinghua Technology Co., Ltd.), JW-3021HR centrifuge (Anhui Jiawen), JS-1070p automatic exposure instrument (Shanghai Peiqing Technology Co., Ltd.), GL-88B vortex mixer (Qilinbei Instrument Manufacturing Company), K960 PCR instrument (Hangzhou Jingle Scientific Instrument Co., Ltd.), MINI-P25 microplate minicentrifuge (Hangzhou Aosheng Instrument Co., Ltd.), LX300 low-speed minicentrifuge (Qilinbei Instrument Manufacturing Company), EPS300 electrophoresis instrument (Shanghai Tanon Technology Co., Ltd.), PIKOREAL 96 fluorescent quantitative PCR instrument (Thermo Scientific), 10212432C PIKO Plate Illuminator (Thermo Scientific), OD1000+ ultra-microspectrophotometer (Nanjing Wuyi Technology Co., Ltd.), VE-180 electrophoresis tank (Shanghai Tanon Technology Co., Ltd.), a VE-186 film transfer instrument (Shanghai Tanon Technology Co., Ltd.), and pH metre (Shanghai Mettler Toledo instrument Co., Ltd.).

The article "Effect of Acupuncture on Simple Obesity and Serum Levels of Prostaglandin E and Leptin in Sprague-Dawley Rats" was published in 2021. Journal: Comput Math Methods Med.

### 2.3. Reagents

The following reagent kits were used: triglyceride test kit (GPO-PAP method) (A035 & 2019007, Changchun Huili Biotechnology Co., Ltd.), high-density lipoprotein cholesterol (direct method-selective inhibition method) (A029 & 2019011, Changchun Huili Biotechnology Co., Ltd.), low-density lipoprotein cholesterol (direct method) (A028 & 2019011 Changchun Huili Biotechnology Co., Ltd.), total cholesterol (A111-1 & 20190515, Nanjing Jiancheng Bioengineering Research Institute), Novostart SYBR qPCR Supermix plus (E096-01B & 0516511, Novoprotein), Primescript™ RT reagent kit with gDNA eraser (RR047A & AJ51485A, TaKaRa), rat high-sensitivity C-reactive protein ELISA Kit (JYM0253Ra & GR2020-06, Wuhan ColorfulGene Technology Co., Ltd.), rat prostaglandin E2 (PGE2) ELISA Kit (JYM0253Ra & GR2020-06, Wuhan ColorfulGene Technology Co., Ltd.), rat leptin ELISA kit (JYM0253Ra & GR2020-06, Wuhan ColorfulGene Technology Co., Ltd.), ECL hypersensitive luminescence kit (34094 & UE283595A, Thermo), goat anti-mouse IgG (ZB-2305 & 140193, Zsbio), and goat anti-rabbit IgG (ZB-2301 & 206820103, Zsbio). The primers were synthesized by SANGON Biotechnology.

### 2.4. Animal Experiment and Grouping

Ten rats were randomly selected and fed a normal diet (12% fat, 3.7% sucrose, Lab Diet 5001). We chose 10 rats at random as the normal group, while we fed the rest a high-fat diet (68% normal diet, 15% sugar, 10% lard, 1% cholesterol, 5% protein powder, 0.8% salt, and 0.2% sodium cholate) for 8 weeks. Rats with body weights greater than 20% of the average body weight of the normal group were used as rat models of simple obesity. The rat models were distributed into two groups: an acupuncture group (study group: 10 rats) and a model group (10 rats).

### 2.5. Acupuncture Intervention Methods

According to the 2016 edition of “Experimental Acupuncture and Moxibustion,” the selected acupoints were punctured at Tianshu 4 mm, Guanyuan 5 mm, Zusanli 3 mm, and Sanyinjiao 4 mm. After obtaining Qi, the G6805-III electroacupuncture instrument was connected, and the density wave was 2-3 mA. We retained the needle for 10 minutes once a day, and the acupoints were selected alternately from left to right for 21 days. The normal group and the model group were fixed for 10 minutes in the same way without acupuncture intervention.

The article "Effect of Acupuncture on Simple Obesity and Serum Levels of Prostaglandin E and Leptin in Sprague-Dawley Rats" was published in 2021. Journal: Comput Math Methods Med.

### 2.6. Experimental Sampling

During the experiment, the body weight and body length (distance from the nose tip to the anal outer edge) were measured at a fixed time every week, and Lee's index was calculated. After the treatment, we fasted the rats for 12 hours but allowed them free access to drinking water. Pentobarbital sodium (2%) was then injected intraperitoneally to anesthetize the rats. We collected blood from the abdominal aorta and separated the serum through centrifugation. The serum levels of leptin, prostaglandin E, CRP, TG, CHO, LDL, HDL, and C-reactive protein were detected. At the same time, the liver was excised and fixed with glutaraldehyde. We observed the morphological changes in the hepatic fat through making use of light and electron microscopy.

### 2.7. Quantitative mRNA Expression Measurement

Use RNeasy Mini Kit (Cat. N 74104, Qiagen) to isolate RNA. Use PrimescriptTM RT reagent kit with gDNA eraser (RR047A & AJ51485A, TaKaRa) to transcribe RNA into cDNA according to manufacturer's protocol. The TaqMan real-time polymerase assay uses Novostart SYBR qPCR Supermix plus (E096-01B & 0516511, Novoprotein). Use PIKOREAL 96 fluorescent quantitative PCR instrument (Thermo Scientific) to amplify and detect thresholds. The target gene expression was normalized to the expression of *β*-actin as a housekeeping gene.

### 2.8. Statistical Analysis

We performed data analysis using SPSS version 20.0 software and expressed the data as the mean ± standard deviation. All experiments were repeated three times. The distributions of continuous data were tested for normality and homogeneity of variance. We analyzed differences in variables by making use of one-way analysis of variance (ANOVA) with LSD or Dunnett's T3 test. We considered differences significant when *P* < 0.05.

## 3. Results

### 3.1. Changes in Body Mass and Lee's Index of Rats in Each Group before and after Treatment

Before treatment, the model group showed normal morphology, decreased activity, and significantly increased body weight in comparison with the normal group. There were no obvious differences in morphology or weight between the acupuncture group and the model group before treatment. The acupuncture group's activity increased, and the weight decreased after acupuncture treatment. As shown in Figures 1 and 2, the body weight and Lee's index of the model group and the acupuncture group before acupuncture treatment were obviously higher than those of the normal group, and there was no obvious difference between the model group and the acupuncture group. After acupuncture treatment, the body weight and Lee's index of the acupuncture group were obviously lower than those of the model group.

The article "Effect of Acupuncture on Simple Obesity and Serum Levels of Prostaglandin E and Leptin in Sprague-Dawley Rats" was published in 2021. Journal: Comput Math Methods Med.

### 3.2. Effects of Acupuncture on Serum Levels of hs-CRP, TG, CHO, LDL, and HDL in Rats of Each Group

From Table 1, we found that the serum levels of hs-CRP, TG, CHO, and LDL in the model group were obviously higher than those in the normal group (*P* < 0.05), while the serum levels of hs-CRP, TG, CHO, and LDL in the acupuncture group were obviously lower than those in the model group (*P* < 0.05). Moreover, the serum level of HDL in the model group was obviously lower than that in the normal group (*P* < 0.05), while the serum level of HDL in the acupuncture group was obviously higher than that in the model group (*P* < 0.05).

### 3.3. Changes in Leptin and Prostaglandin E in Rats of Each Group

As shown in Table 2, the serum level of prostaglandin E in the model group was obviously higher than that in the normal group (*P* < 0.05), and the serum level of prostaglandin E in the acupuncture group was obviously lower than that in the model group (*P* < 0.05). As shown in Figures 3 and 4, the protein and mRNA expression levels of leptin in the model group were obviously higher than those in the normal group (*P* < 0.05), while the protein and mRNA expression levels of leptin in the acupuncture group were obviously lower than those in the model group (*P* < 0.05).

### 3.4. Morphological Changes of Adipose Tissue in Rat Liver

As shown in Figure 5, in the normal group, the liver cells were arranged radially. In the model group, there was obvious inflammation and more fat bubbles in the liver tissue. In comparison with the model group, the degree of inflammation and the number of fat bubbles in the liver tissue of the acupuncture group were obviously decreased. As shown in Figure 6, the liver fat morphology of the model group was obviously larger than that of the normal group, while that of the acupuncture group was obviously smaller than that of the model group.

## 4. Discussion

Obesity is a global epidemic disease that increases the incidence of serious diseases such as type 2 diabetes, cancer, hypertension, nonalcoholic fatty liver disease, cardiovascular diseases, and dementia [13–16]. As for pregnant obese women and their foetus, there is a considerable risk for adverse perinatal outcomes. In morbidly obese women, maternal leptin levels affect foetal development, birth weight, and the growth trajectory of lactation [17–19]. Obesity has been identified as a cause of esophageal cancer, colon cancer, uterine cancer, kidney cancer, and postmenopausal breast cancer. It is also an important risk factor for prostate cancer, pancreatic cancer, and non-Hodgkin's lymphoma [20]. Therefore, revealing the regulation of obesity by acupuncture is of great significance to human health.

The article "Effect of Acupuncture on Simple Obesity and Serum Levels of Prostaglandin E and Leptin in Sprague-Dawley Rats" was published in 2021. Journal: Comput Math Methods Med.

CRP is considered to be a key plasma protein that can bind to leptin [21]. Studies have shown that CRP is positively correlated with increased body mass index [22]. Mammals store metabolic energy in the form of TG in adipose tissue [23]. Metabolic cardiomyopathy (MC) is characterized by the accumulation of TG and lipotoxic damage in the myocardium, which is a new cause of heart failure in obese patients [24]. Elevated LDL is a treatable and heritable risk factor for cardiovascular disease. Obesity is an important risk factor for various chronic diseases. It is generally related to dyslipidemia. It is mainly manifested as a decrease in HDL, which plays an indispensable role in the development of cardiovascular diseases [25]. In this study, the serum hs-CRP, TG, CHO, and LDL levels of the model group were significantly higher than those of the normal group, while the serum hs-CRP, TG, CHO, and LDL levels of the acupuncture group were significantly lower than those of the model group. The serum HDL of the model group was significantly lower than that of the normal group, while the HDL of the acupuncture group was significantly higher than that of the model group. In summary, acupuncture effectively regulates SD-related markers.

Simple obesity is a metabolic disease with a complex etiology. Leptin and leptin resistance are closely related to the occurrence and development of simple obesity [26]. The serum leptin level was positively correlated with the body mass index (BMI) [27]. In the case of obesity, a decrease in plasma leptin levels can restore hypothalamic leptin sensitivity and effectively reduce weight gain [28]. Inflammation of white adipose tissue has a crucial influence on the development of obesity. Prostaglandin E2 (PGE2) is involved in lipolysis and adipogenesis. In this study, the serum prostaglandin e levels, leptin protein, and mRNA expression levels in the model group were significantly higher than those in the normal group. This is consistent with previous reports that obesity leads to increased prostaglandin e and leptin protein levels. In addition, the levels of prostaglandin e, leptin protein, and mRNA expression in the acupuncture group were significantly lower than those in the model group. Acupuncture can improve leptin resistance, promote leptin receptor gene expression, inhibit NPY gene expression, and activate the leptin signaling pathway and other ways to achieve weight loss [29]. Meanwhile, acupuncture can also significantly improve the blood lipid status and reduce the expression of inflammatory factors [30]. Acupuncture may reduce the expression levels of prostaglandin e and leptin to regulate obesity.

The article "Effect of Acupuncture on Simple Obesity and Serum Levels of Prostaglandin E and Leptin in Sprague-Dawley Rats" was published in 2021. Journal: Comput Math Methods Med.

There are still some limitations in this study. First of all, it is necessary to further explore the exact mechanism of acupuncture regulating obesity. Secondly, the regulatory pathways of acupuncture at different acupoints on simple obesity are still unclear. In future research, we will conduct this exploration.

In conclusion, this study explored the effect and mechanism of acupuncture in the treatment of simple obesity. Acupuncture significantly reduced serum CRP, TG, CHO, LDL, leptin, and prostaglandin E levels in simple obese rats and increased HDL levels. This study further confirms the role of acupuncture in weight loss and provides new direction and supporting evidence for other researchers' investigations.

## Figures and Tables

**Figure 1:** The effect of acupuncture on the body weight of Sprague-Dawley rats. ^∗^*P* < 0.05.

**Figure 2:** The effect of acupuncture on Lee's index of Sprague-Dawley rats. ^∗^*P* < 0.05.

**Figure 3:** Leptin's protein expression level in each group.

**Figure 4:** Leptin's mRNA expression level in each group. ^∗^*P* < 0.05.

**Figure 5:** The morphology of adipose tissue in rat liver was observed by light microscope.

**Figure 6:** We observed the morphology of adipose tissue in rat liver through making use of an electron microscope.

**Table 1:** Serum levels of hs-CRP, TG, CHO, LDL, and HDL in each group.

	Normal group	Model group	Acupuncture group
hs-CRP	6791.78 ± 125.38	9333.42 ± 122.45^∗^	8581.68 ± 180.63^#^
TG	2.11 ± 0.06	2.59 ± 0.05^∗^	2.44 ± 0.06^#^
CHO	3.86 ± 0.15	5.86 ± 0.26^∗^	4.44 ± 0.16^#^
LDL	2.15 ± 0.05	2.44 ± 0.05^∗^	2.29 ± 0.03^#^
HDL	1.51 ± 0.05	1.14 ± 0.04^∗^	1.29 ± 0.05^#^

Compared with the normal group, ^∗^*P* < 0.05; compared with model group, ^#^*P* < 0.05.

**Table 2:** TG and serum levels of leptin and PGE2 in each group.

	Normal group	Model group	Acupuncture group
Leptin	952.37 ± 164.72	2560.41 ± 248.39^∗^	1255.95 ± 146.62^#^
PGE2	43.48 ± 6.88	112.92 ± 10.41^∗^	69.26 ± 12.24^#^

Compared with normal group, ^∗^*P* < 0.05; compared with model group, ^#^*P* < 0.05.

## Data Availability

The datasets used and/or analyzed during the current study are available from the corresponding author on reasonable request.

## References

[1] Gellner R., Domschke W. (2008). Epidemiology of obesity. *Der Chirurg; Zeitschrift fur alle Gebiete der operativen Medizen*.

[2] Kolovou G. D., Watts G. F., Mikhailidis D. P. (2019). Postprandial hypertriglyceridaemia revisited in the era of non-fasting lipid profile testing: a 2019 expert panel statement. *Current vascular pharmacology*.

The article "Effect of Acupuncture on Simple Obesity and Serum Levels of Prostaglandin E and Leptin in Sprague-Dawley Rats" was published in 2021. Journal: Comput Math Methods Med.

[3] Nguyen D. M., El-Serag H. B. (2010). The epidemiology of obesity. *Gastroenterology Clinics of North America*.

[4] Lee Y., Lee K. S. (2019). Relationship between unhealthy weight control behaviors and substance use patterns among Korean adolescents: results from the 2017 national youth risk behavior survey. *Public Health*.

[5] Kirk S. F., Penney T. L., McHugh T. L., Sharma A. M. (2012). Effective weight management practice: a review of the lifestyle intervention evidence. *International Journal of Obesity*.

[6] Powell L. H., Calvin J. E., Calvin J. E. (2007). Effective obesity treatments. *The American Psychologist*.

[7] Wirth A., Wabitsch M., Hauner H. (2014). The prevention and treatment of obesity. *Deutsches Ärzteblatt International*.

[8] Qunli W., Zhicheng L. (2005). Acupuncture treatment of simple obesity. *Journal of Traditional Chinese Medicine*.

[9] Kaptchuk T. J. (2002). Acupuncture: theory, efficacy, and practice. *Annals of Internal Medicine*.

[10] Acar H. V. (2016). Acupuncture and related techniques during perioperative period: a literature review. *Complementary Therapies in Medicine*.

[11] Wang L., Yu C. C., Li J., Tian Q., Du Y. J. (2021). Mechanism of action of acupuncture in obesity: a perspective from the hypothalamus. *Frontiers in Endocrinology*.

[12] Shu Q., Chen L., Wu S. (2020). Acupuncture targeting SIRT1 in the hypothalamic arcuate nucleus can improve obesity in high-fat-diet-induced rats with insulin resistance via an anorectic effect. *Obesity Facts*.

[13] Shin M. K., Eraso C. C., Mu Y. P. (2019). Leptin induces hypertension acting on transient receptor potential melastatin 7 channel in the carotid body. *Circulation Research*.

[14] Pena-Cano M. I., Saucedo R., Morales-Avila E., Valencia J., Zavala-Moha J. A., Lopez A. (2019). Deregulated microRNAs and adiponectin in postmenopausal women with breast cancer. *Gynecologic and Obstetric Investigation*.

[15] Smith P. J., Mabe S., Sherwood A. (2019). Association between insulin resistance, plasma leptin, and neurocognition in vascular cognitive impairment. *Journal of Alzheimer's disease: JAD*.

[16] Telschow A., Ferrari N., Deibert C. (2019). High maternal and low cord blood leptin are associated with BMI-SDS gain in the first year of life. *Obesity Facts*.

[17] Serapio S., Ahlsson F., Larsson A., Kunovac Kallak T. (2019). Second trimester maternal leptin levels are associated with body mass index and gestational weight gain but not birth weight of the infant. *Hormone Research in Pædiatrics*.

The article "Effect of Acupuncture on Simple Obesity and Serum Levels of Prostaglandin E and Leptin in Sprague-Dawley Rats" was published in 2021. Journal: Comput Math Methods Med.

[18] Arroyo-Jousse V., Jaramillo A., Castano-Moreno E., Lepez M., Carrasco-Negue K., Casanello P. (2020). Adipokines underlie the early origins of obesity and associated metabolic comorbidities in the offspring of women with pregestational obesity. *Biochimica et Biophysica Acta - Molecular Basis of Disease*.

[19] Zamanillo R., Sanchez J., Serra F., Palou A. (2019). Breast milk supply of microRNA associated with leptin and adiponectin is affected by maternal overweight/obesity and influences infancy BMI. *Nutrients*.

[20] Wolin K. Y., Carson K., Colditz G. A. (2016). Obesity and cancer. *The Oncologist*.

[21] Sudhakar M., Silambanan S., Chandran A. S., Prabhakaran A. A., Ramakrishnan R. (2018). C-reactive protein (CRP) and leptin receptor in obesity: binding of monomeric CRP to leptin receptor. *Frontiers in Immunology*.

[22] Khaodhiar L., Ling P. R., Blackburn G. L., Bistrian B. R. (2004). Serum levels of interleukin-6 and C-reactive protein correlate with body mass index across the broad range of obesity. *JPEN Journal of Parenteral and Enteral Nutrition*.

[23] Frayn K. N., Arner P., Yki-Jarvinen H. (2006). Fatty acid metabolism in adipose tissue, muscle and liver in health and disease. *Essays in Biochemistry*.

[24] Costantino S., Akhmedov A., Melina G. (2019). Obesity-induced activation of JunD promotes myocardial lipid accumulation and metabolic cardiomyopathy. *European Heart Journal*.

[25] Carroll K. K. (1998). Obesity as a risk factor for certain types of cancer. *Lipids*.

[26] Oh S., Son M., Choi J. (2019). Phlorotannins from *Ecklonia cava* attenuates palmitate-induced endoplasmic reticulum stress and leptin resistance in hypothalamic neurons. *Marine drugs*.

[27] Osateerakun P., Weerasopone S., Amarase C., Honsawek S., Limpaphayom N. (2019). Serum adipokine levels, bodyweight and functional status in children with cerebral palsy. *Obesity Medicine*.

[28] Mzhelskaya K. V., Shipelin V. A., Shumakova A. A. (2020). Effects of quercetin on the neuromotor function and behavioral responses of Wistar and Zucker rats fed a high-fat and high-carbohydrate diet. *Behavioural Brain Research*.

[29] Schwartz M. W., Baskin D. G., Bukowski T. R. (1996). Specificity of leptin action on elevated blood glucose levels and hypothalamic neuropeptide Y gene expression in *ob/ob* mice. *Diabetes*.

[30] Chen Y., Huang W., Li Z. (2019). The effect of acupuncture on the expression of inflammatory factors TNF-*α*, IL-6,IL-1 and CRP in cerebral infarction. *Medicine (Baltimore)*.

